The article "Difference between Mechanical Alignment in Navigation and Scanogram during Total Knee Arthroplasty" was retracted in 2020. Reasons: errors in the data; errors in the methods.

# Difference between Mechanical Alignment in Navigation and Scanogram during Total Knee Arthroplasty

**DOI:** 10.1155/2019/4096306

**Published:** 2019-04-01

**Authors:** Rohan Bhimani, Fardeen Bhimani, Preeti Singh

**Affiliations:** ^1^Department of Orthopaedics, Hinduja Healthcare Surgical, 11^th^ Road, Khar West, Mumbai 400052, India; ^2^Department of Orthopaedics, Bharati Hospital, Pune 411043, India; ^3^Department of Orthopaedics, Osmania General Hospital, Hyderabad 500012, India

## Abstract

**Introduction:**

Malpositioning of the implant results in polyethylene wear and loosing of implant after total knee arthroplasty. Scanogram is often used for measurement of limb alignment. Computer navigation provides real time measurements and thus, the aim is to see any association pre- and postoperatively between coronal alignments measured on scanogram to computer navigation during total knee arthroplasty.

**Material and Methods:**

We prospectively gathered data of 200 patients with advanced degenerative symptomatic arthritis, who were consecutively selected for primary total knee arthroplasty with computer navigation. Every patient's pre- and postoperative scanogram were compared to the intraoperative computer navigation findings.

**Results:**

The results show that the preoperative mean mechanical axis on navigation was 10.65° (SD ± 6.95) and on scanogram it was 10.38° (SD ± 6.89). On the other hand, the mean postoperative mechanical axis on navigation was 0.69° (SD ± 0.87) and on scanogram it was 2.73° (SD ± 2.10). Preoperatively, there was no significant difference (p value = 0.46) between the two. However, the postoperative outcomes suggest that there was a noteworthy difference, with no correlation between the mean Hip-Knee Ankle Axis (HKA) and intraoperative mechanical axis (p value <0.0001).

**Conclusion:**

Postoperative mechanical alignment values after total knee arthroplasty are lower on navigation than measured on standing full length hip to ankle scanogram.

## 1. Introduction

Reinstatement of the mechanical axis of the knee is one of the key parameters for long term success in total knee arthroplasty. Misalignment more than 3° (varus or valgus) increases the rate of polyethylene wear and consequent loosening in total knee arthroplasty (TKA) [1]. For TKA to be successful, precise preoperative planning, intraoperative application, and postoperative evaluation by accurate measurements of coronal alignment of the lower limb are important. For assessing this alignment various techniques like scanogram, CT scan, etc. are available. Of these, scanogram is considered the gold standard as it takes into consideration the competence of the ligaments in weight bearing orientation of the limb [1–4]. But the chief drawback of scanogram is that it does not take into consideration the third dimension of the limb and thus for accuracy, the scanogram should be taken in the plane of measurement.

The article "Difference between Mechanical Alignment in Navigation and Scanogram during Total Knee Arthroplasty" was retracted in 2020. Reasons: errors in the data; errors in the methods.

The introduction of computer navigation has helped surgeons with real time images and to achieve measurements within 1°, which are accurate and reproducible [5–8]. This system registers the bony landmarks by direct contact and assists with precise calculation, correction of alignment, and component placement during the surgery.

The purpose of this study is to see any association pre- and postoperatively between coronal alignments measured on scanogram to that by computer navigation during total knee arthroplasty. The authors have hypothesized a positive correlation, pre- and postoperatively, in the mechanical alignment of the lower limb between scanogram and navigation system findings.

## 2. Materials and Methods

### 2.1. Patient Selection

Between October 2016 and December 2017, 200 patients with advanced degenerative symptomatic arthritis were consecutively selected for primary total knee arthroplasty with computer navigation. We prospectively gathered their data. The exclusion criteria included previous knee surgery and frontal plane deformity greater than 25°. There were 89 males and 111 females with the mean age of 65 (range 49 to 81 years). All patients gave written consent to be a part of the study.

### 2.2. Pre-Op Planning

All patients preoperatively underwent scanogram, i.e., full length hip to ankle x-ray in weight bearing position. The anteroposterior roentgenogram was taken with feet apart equal to shoulder width, patella facing forward, and knee in maximum extension. The x-ray beams were focused at the level of joint line and the lower limb mechanical axis was then calculated on digitally processed scanogram. The hip-knee-ankle (HKA) angle was measured from the centre of femoral head to the centre of the knee and from there to the centre of the ankle. Positive angles indicate varus and negative angles indicate valgus. All scanograms were evaluated and were retaken if found in inappropriate position or poor quality.

### 2.3. Surgical Technique

Surgeries were performed either under spinal anaesthesia for unilateral total knee arthroplasty or under combined spinal and epidural anaesthesia for bilateral cases. Conventional anterior midline skin incision followed by medial parapatellar arthrotomy was carried out. Posterior cruciate ligament resection and patellar resurfacing were done in all cases. The navigation system of image-free Ci Navigation System (Brainlab AG, Munich, Germany) was used to record intraoperative mechanical axis. The external tracking arrays were placed on distal femur and proximal tibia using screws. Various anatomical landmarks such as medial and lateral epicondyle, medial malleolus, lateral malleolus, central point of ankle, and medial and lateral point of tibial plateau were recorded using pointer device which provided data to the infrared receiver and real time images were displayed both in frontal and in sagittal plane. Proximal tibial cut followed by distal femur cut was made. Tensioner assisted ligament balancing was performed. Under navigation guidance, flexion and extension gaps were balanced. After navigation assisted cuts were taken, the trial component and spacer were placed next and knee R.O.M. was assessed. We used PFC Sigma implants (Depuy orthopaedic, Warsaw, IN, USA). Next the final cement component placement was carried out, and the final mechanical axis was checked on the navigation system after reducing the patella and before closing the fascia. Lastly patellar tracking and knee range of movements were clinically assessed and closure of wound was carried out followed by application of jones bandage.

The article "Difference between Mechanical Alignment in Navigation and Scanogram during Total Knee Arthroplasty" was retracted in 2020. Reasons: errors in the data; errors in the methods.

### 2.4. Post-Op Management

The day following the surgery, isometric quadriceps, active ankle, straight leg raises, and knee bending exercises were started. As per our protocol, full length hip to ankle standing scanogram were performed on all patients before discharge. The mechanical alignment of the lower limb was calculated on these scanograms. Finally, the correlations between navigation and pre- and postoperative scanogram alignments were analysed.

### 2.5. Statistical Analysis

The test was used to compare the pre- and postoperative measured alignments between scanogram and computer navigation. Statistical data analysis was conducted using SPSS 18.0. Student t-test and chi square test were used to compare the level of significance with p value ≤0.05 considered as statistically significant.

## 3. Results

The mean preoperative and postoperative mechanical axis on navigation and scanogram are mentioned in Table 1. The preoperative mean mechanical axis on navigation was 10.65° (SD ± 6.95) and on scanogram was 10.38° (SD ± 6.89). The mean of the difference in the preoperative mechanical axis values was 0.27° (SD ± 0.06). On the other hand, the mean postoperative mechanical axis on navigation was 0.69° (SD ± 0.87) and on scanogram was 2.73° (SD ± 2.10). The mean of the difference in the postoperative mechanical axis was 2.04° (SD ± 1.23).

Initial preoperative navigation and scanogram measurements showed large degrees of deformity, but their mean values and standard deviation were similar. The preoperative Bland-Altman plot (Figure 1) shows a tendency for varus knee (right-hand side of plot) to be in bottom quadrant with the limit of agreement between 1.60 and 6.86. The final navigation value and postoperative scanogram measurements were reduced but their mean value and standard deviation were not similar and had a difference of 2.04° in their mean values. The postoperative Bland-Altman plot shows varus knee (right-hand side of plot) and an upward linear trend with limit of agreement between -1.41 and 6.14 (Figure 2).

The article "Difference between Mechanical Alignment in Navigation and Scanogram during Total Knee Arthroplasty" was retracted in 2020. Reasons: errors in the data; errors in the methods.

According to our hypothesis, we aimed to determine if there was correlation between alignment determined on scanogram and navigation. The trends indicated that there was correlation preoperatively with no significant difference (p value = 0.42). However, the postoperative trends suggest that there was a significant difference, with no correlation between the mean HKA and intraoperative mechanical axis (p value <0.0001). Furthermore, 25% of the outliers showed a difference of >3° between the mechanical axis on navigation at the end of total knee arthroplasty and the postoperative HKA measurements as shown in Figure 3.

## 4. Discussion

This study analyses whether limb mechanical alignment achieved by navigation during total knee arthroplasty correlates with alignment measured on scanogram. We found that computer navigation assisted limb alignment correlated with preoperative scanogram alignment findings but not with postoperative scanogram alignment measurements. In spite of the fact that precise correction of lower limb alignment is an essential factor for TKA, it is not easy to achieve [9].

N.M.J. Wilcox et al. [5] assessed the relationship between radiological and navigation measurements of lower limb and observed that preoperative mechanical alignment on long leg radiograph was varus of 3.6° ± 8.9 and on navigation was varus of 3.3° ± 6.4. These two sets of measurements showed moderate correlation (p = 0.275). In the current study, we observed varus of 10.38° ± 6.89 on preoperative scanogram and 10.65° ± 6.95 on preoperative navigation. The findings correlated well and there was no significant difference (p = 0.46).

Sina Babazadeh et al. [10] compared long leg radiograph to computer navigation for assessing alignment postoperatively. They found that correlation between long leg radiograph and intraoperative navigation was 0.614 (p < 0.0001). Another similar study by Won Chul Choi et al. [7] showed postoperative mechanical alignment varus of 0.3° ± 2.9 on long leg radiograph and 0.1° ± 1.2 on navigation, with no correlation between the two measurements (p = 0.310). In our study, we observed that postoperative alignment was 2.73° ± 2.10 varus on scanogram and 0.69° ± 0.87 varus on navigation. There was no correlation between these findings and trends suggested a significant difference between the two measurements (p < 0.0001). The number of outliers accounted for 25%, having difference of > 3° on navigation and scanogram measurements.

The article "Difference between Mechanical Alignment in Navigation and Scanogram during Total Knee Arthroplasty" was retracted in 2020. Reasons: errors in the data; errors in the methods.

A few studies in the past have shown that navigation TKA are more accurate than long leg radiographs at controlling intraoperative alignment [7]. But, this has not been taken as a gold standard. On the contrary, many studies have postulated that postoperative scanograms are more reliable in measuring coronal plane alignment as compared to navigation system [6, 10]. The disagreement between navigation and scanogram alignments is due to their respective limitations. The axis on computer navigation is determined by calculation based on anatomical landmarks. Inter- as well as intrasurgeon variation for noting these landmarks may be one of the causes of disagreement. Additionally, measurements on navigation are made without taking weight bearing into consideration and with fascia open which affects the alignment. Various factors like limb rotation, flexion contracture, muscle tone, weight bearing, and antalgic stance affect measurements on scanogram. The inaccuracy escalates with rotation of leg and flexion contracture. The difference of measured limb alignment of up to 4° has been observed due to various combinations of flexion and rotations [1]. In addition to this, the weight bearing scanogram also takes into consideration soft tissue tension and ligament imbalance leading to disparity between measurements. The muscle tone which is absent under anaesthesia also has an effect on scanogram.

Robert Karl Zahn et al. [11] showed that immediate postoperative standing long leg radiograph is of limited value because limb loading is altered because of antalgic component and is therefore nonphysiological. The actual coronal alignment should be assessed at physiological loading.

The current study has some limitations. The scanogram alignment was measured and analysed immediately postoperatively during hospital stay. A longer follow-up may influence the mechanical alignment variations in form of loss of correction, improvement of remaining flexion contracture, and decrease in antalgic component. In addition, errors can occur due to faulty and inconsistent radiographic techniques. We minimized these errors by using standard scanogram protocol.

## 5. Conclusion

Postoperative mechanical alignment values after total knee arthroplasty are lower on navigation than measured on standing full length hip to ankle scanogram.

## Figures and Tables

**Figure 1:** Bland-Altman plot showing relation between difference and mean of preoperative values of alignment.

The article "Difference between Mechanical Alignment in Navigation and Scanogram during Total Knee Arthroplasty" was retracted in 2020. Reasons: errors in the data; errors in the methods.

**Figure 2:** Bland-Altman plot demonstrating relation between difference and mean of postoperative values of alignment.

**Figure 3:** Categorized distribution of difference in mechanical alignment of navigation and scanogram postoperatively.

**Table 1:** Measured Limb Alignment on Navigation and Scanogram.

	Mean	Standard Deviation	Mean of the Difference	Standard Deviation of Difference	P Value
Pre-Op Mechanical Axis On Navigation	10.65°	6.95°	0.27°	0.06°	0.42
Pre-Op Mechanical Axis On Scanogram	10.38°	6.89°			

Post-Op Mechanical Axis On Navigation	0.69°	0.87°	2.04°	1.23°	<0.0001
Post-Op Mechanical Axis On Scanogram	2.73°	2.10°			

## Data Availability

All data generated or analyzed during this study are included in this article.
